# Early venous thromboembolism at the beginning of palliative chemotherapy is a poor prognostic factor in patients with metastatic pancreatic cancer: a retrospective study

**DOI:** 10.1186/s12885-018-5154-3

**Published:** 2018-12-17

**Authors:** Jung Sun Kim, Eun Joo Kang, Dae Sik Kim, Yoon Ji Choi, Suk Young Lee, Hong Jun Kim, Hee Yeon Seo, Jun Suk Kim

**Affiliations:** 1 Division of Hematology/Oncology, Department of Internal Medicine, Korea University College of Medicine, 148 Gurodong-ro, Guro-gu, Seoul, 08308 South Korea; 2 Division of Hematology/Oncology, Department of Internal Medicine, Korea University College of Medicine, 148 Gurodong-ro, Guro-gu, Seoul, 08308 South Korea; 3 Division of Hematology/Oncology, Department of Internal Medicine, Konkuk University School of Medicine, Chungchungbukdo, Chungju, South Korea

**Keywords:** Pancreatic cancer, Venous thromboembolism, Prognosis, Predictive value, Chemotherapy, Khorana score, Hyponatremia

## Abstract

**Background:**

This study investigated the prognostic effects of venous thromboembolism (VTE)-related factors in patients with metastatic pancreatic cancer receiving palliative chemotherapy. Predictive factors for VTE were also investigated.

**Methods:**

A total of 216 patients diagnosed with metastatic pancreatic cancer who received gemcitabine-based palliative chemotherapy at our institution were retrospectively evaluated.

**Results:**

VTE occurred in 51 (23.6%) patients during treatment and did not affect survival. However, patients who were diagnosed with VTE at the beginning of chemotherapy showed poor prognosis compared with patients diagnosed with VTE during chemotherapy: all patients (hazard ratio [HR] 1.897, *p* = 0.008); patients diagnosed with VTE (HR = 3.768, *p* = 0.001). Low serum sodium (Na) (< 135 mmol/L) and high Khorana score (≥3) were strong predictive factors of early VTE (odds ratio [OR] 5.109; 95% confidence interval [95% CI] = 1.010–25.845; *p* = 0.049 for Khorana score, OR 10.304; 95% CI = 1.036–102.466; *p* = 0.047) for hyponatremia).

**Conclusions:**

Our study demonstrated that occurrence and detection of VTE in the early period of chemotherapy was the most significant VTE-related prognostic factor in patients with metastatic pancreatic cancer receiving chemotherapy. Prediction using the Khorana score and serum Na levels would be helpful in early diagnosis of VTE.

## Background

Pancreatic cancer is a highly lethal malignancy and a major cause of cancer-related death. The incidence of pancreatic cancer continues to increase worldwide, but improvements in patient survival have been dismal. The median overall survival (OS) of patients with unresectable metastatic pancreatic cancer without treatment is less than 4 months [1]. Despite significant developments in systemic treatment for patients with advanced pancreatic cancer, most patients survive less than 1 year and the 5-year survival rate is less than 10% [2].

Cancer is a well-known risk factor for venous thromboembolism (VTE). The risk of VTE is 4- to 7-fold higher in patients with cancer compared to patients without cancer [3]. Among various cancer types, pancreatic cancer is associated with the highest risk of VTE occurrence [4]. Moreover, chemotherapy further increases the risk of VTE [5]. Therefore, patients with advanced pancreatic cancer receiving chemotherapy are at very high risk of VTE.

The characteristics of cancer-related VTE in terms of anatomical site, symptoms, and complications differ widely. VTE is fatal in some patients, while others experience no discomfort associated with VTE during cancer treatment. In general, cancer-related VTE leads to poor survival in patients with cancer [6]. However, specific VTE-related factors that significantly affect prognosis have not been identified in patients with advanced pancreatic cancer. Furthermore, predictors for significant VTE-related factors that might affect survival are currently unknown in this population. In actual clinical practice, oncologists should determine appropriate anticoagulation treatment in patients according to whether VTE occurred before or during chemotherapy. Anticoagulant therapy may have fatal side effects such as bleeding, which can interrupt cancer treatment and lead to mortality. Decisions regarding anticoagulant therapy are difficult even when patients are diagnosed with VTE; thus, anticoagulation treatment should be provided based on individual patient characteristics. Information regarding prognostic VTE-related factors and predictors would assist oncologists in predicting the occurrence of VTE and in determining active cancer treatment as well as anticoagulant therapy in clinical practice.

The efficacy of prophylactic anticoagulation in patients at high risk for VTE is also under debate. In previous clinical trials, routine thromboprophylaxis in patients with pancreatic cancer receiving chemotherapy did not improve survival outcomes, although primary thromboprophylaxis decreased the incidence of VTE [7]. Therefore, routine thromboprophylaxis is not recommended for all patients with pancreatic cancer, even those at very high risk of VTE [8, 9]. Additional investigation is thus required to identify a subgroup of patients among all of those at high-risk of VTE for whom thromboprophylaxis may be beneficial.

Therefore, in the present study, we attempted to identify particular characteristics of VTE that are associated with poor survival in patients with metastatic pancreatic cancer receiving palliative chemotherapy. We also attempted to identify clinical factors to predict patients with VTE-related risk factors that can be related to poor survival.

## Methods

### Patients and methods

The medical records of patients with pancreatic cancer diagnosed at the Korea University Guro Hospital between January 2005 and December 2015 were reviewed. Among the patients identified, those with inoperable, recurrent, or metastatic pancreatic cancer who received palliative chemotherapy were consecutively included in this retrospective study. Baseline and clinical data from the time of initial cancer diagnosis until December 31, 2016 were retrieved.

Electronic medical records of patients were reviewed, and the clinical information for each patient, including demographic data, body mass index (BMI), body surface area (BSA), history of diabetes mellitus (DM), site of primary mass, previous surgery, Eastern Cooperative Oncology Group Performance Status (ECOG PS), treatment history, laboratory findings at the beginning of chemotherapy, and VTE occurrence, were investigated. Measurement of inflammatory markers, such as the neutrophil-to-lymphocyte ratio (NLR) and platelet-to-lymphocyte ratio (PLR), prior to the initiation of chemotherapy, were also examined. In addition, we focused on variables included in Khorana’s predictive model and calculated the Khorana score, which is a popular tool for VTE risk prediction in patients with cancer receiving chemotherapy [4]. According to Khorana’s model, pancreatic cancer is associated with a significantly high risk for VTE development, with a base score of 2. In addition, pre-chemotherapy platelet (PLT) count > 350,000/μL and white blood cell (WBC) count > 11,000/μL, hemoglobin (Hb) level < 10 g/dL, use of red cell growth factors, and BMI ≥35 kg/m^2^ are significant risk factors, with each corresponding to a score of 1 in Khorana’s predictive model. Regarding BMI, the number of patients with values ≥35 kg/m^2^ or higher among Asian patients with pancreatic cancer were expected to be very low. In this study, only one patient had a BMI in this range; therefore, we reduced the cut-off to ≥30 kg/m^2^, which is regarded as a criterion for obesity. We were unable to compare the use of red cell growth factors, because all patients included in this study were not prescribed red cell growth factors during chemotherapy. According to Khorana’s model, patients with a score > 3 were classified as high-risk, while those with a score of 2 were classified as the intermediate-risk group.

### Venous thromboembolism diagnosis

To collect information regarding VTE occurrence, computed tomography (CT) and magnetic resonance imaging (MRI) scans of the chest, abdomen and pelvis, extremities, and brain and ultrasonography scans of the extremities were reviewed. If patient was suspected to have VTE, lower extremity CT venography and/or CT pulmonary angiography was performed. From these imaging results, all VTE events including deep vein thrombosis (DVT), pulmonary embolism (PE), visceral venous thrombosis (VVT), and central venous catheter-related thrombosis were collected. Because serial chest, abdomen, and pelvic CT were performed on all patients at around 6–8 weeks intervals during chemotherapy, we could obtain complete information regarding VTE such as detection day; location; and symptom presence, existence, and disappearance. Because early onset or synchronous VTE with cancer can affect whole cancer prognosis, treatment and quality of life, we divided patients into early VTE and late VTE group and analyzed. Patients diagnosed with VTE within 30 days from the start of palliative chemotherapy were assigned to the early VTE group, whereas those diagnosed with VTE at least 30 days after the beginning of palliative chemotherapy were assigned to the late VTE group. Information regarding the presence of symptoms and treatments for VTE was obtained through electronic medical records. This study was approved by the Institutional Review Board of the Korea University Guro Hospital (KUGH 16320–001).

### Statistical analysis

Associations between characteristics of patients with or without VTE were investigated using the Chi-square test. The prognostic effect of VTE on survival was also analyzed. Survival was calculated using the Kaplan-Meier method. OS from chemotherapy was defined as the time from the beginning of palliative chemotherapy for pancreatic cancer to death from any cause. OS from VTE was defined as the time from VTE diagnosis to death from any cause. Comparisons between different characteristics were made using the log-rank test. To evaluate the impact of VTE occurrence on OS and to investigate independent prognostic factors, (variables with *p* < 0.05) we investigated using the time-dependent covariate multiple Cox model. Also, Cox proportional hazard model was used to evaluate the impact of early VTE on OS and to investigate independent prognostic factors. Moreover, associations between characteristics of patients with or without synchronous VTE were investigated using the Chi-square test. Multivariate logistic regression was performed with variables that showed significance using the Chi-square test. All statistical analyses were performed using IBM SPSS Statistics for Windows, version 21.0 (IBM Corp., Armonk, NY, USA).

## Results

### Patient characteristics

Of the 326 patients with pancreatic cancer who received palliative chemotherapy at our institution, data for 216 patients with metastatic pancreatic cancer were retrieved and analyzed. The median age of the patients included in the study was 63 years (range, 38–83).

All patients received gemcitabine alone or gemcitabine-based combination chemotherapy as the first-line treatment: gemcitabine only (8.3%), gemcitabine + erlotinib (35.2%), gemcitabine + fluorouracil (capecitabine, TS-1, or tegafur/uracil 46.3%), gemcitabine + platinum (oxaliplatin or carboplatin, 1.4%), gemcitabine + nab-paclitaxel (0.5%), gemcitabine +/− clinical trial agents included in phase III studies (8.3%).

Of the 216 patients, 51 (23.6%) experienced VTE during treatment courses. Characteristics of all patients and comparison of the characteristics of patients with and without VTE are shown in Table 1. The characteristics of patients with and without VTE were not significantly different.

**Table 1:** Characteristics of patients (*N* = 216)

	No VTE		VTE		Total	*P-value*
	*N*	%	*N*	%	*N*	
Age, median (range)						
< 70 years	113	75.3	37	24.7	150	0.425
≥ 70 years	53	80.3	13	19.7	66	
Sex						
Male	108	82.4	23	17.6	131	0.016
Female	58	68.2	27	31.8	85	
BSA						
< 1.8 m^2^	153	78.1	43	21.9	196	0.187
≥ 1.8 m^2^	13	65	7	35	20	
BMI						
< 30 kg/m^2^	162	77.1	48	22.9	210	0.549
≥ 30 kg/m^2^	4	66.7	2	33.3	6	
DM						
No	90	73.2	33	26.8	123	0.14
Yes	76	81.7	17	18.3	93	
Site of primary mass:						
Head	80	79.2	21	20.8	101	0.506
Body	28	80	7	20	35	
Tail	58	72.5	22	27.5	80	
Previous surgery:						
Palliative	10	83.3	2	16.7	12	0.584
None	156	76.5	48	23.5	204	
ECOG PS						
0–1	150	76.5	46	23.5	196	0.726
2–3	16	80	4	20	20	
WBC						
< 11,000/μL	136	75.1	45	24.9	181	0.174
≥ 11,000/μL	30	85.7	5	14.3	35	
Hb						
< 10 g/dL	31	68.9	14	31.1	45	0.404
≥ 10 g/dL	193	74.8	65	25.2	258	
PLT						0.091
< 350,000/μL	148	78.7	40	21.3	188	
≥ 350,000/μL	18	64.3	10	35.7	28	
CA19–9						
< 1000 U/mL	88	75.2	29	24.8	117	0.535
≥ 1000 U/mL	78	78.8	21	21.2	99	
Khorana score						
Intermediate–risk (2)	105	77.8	30	22.2	135	0.677
High-risk (≥3)	61	75.3	20	24.7	81	
CVC insertion						
No	32	69.6	14	30.4	46	0.219
Yes	133	78.2	37	21.8	170	
Chemotherapy more than first-line						
≥ Second-line	68	81	16	19	84	0.205
First-line only	88	72.7	33	27.3	121	
Unknown	10	90.9	1	9.1	11	
Number of metastatic organs						
< 3	40	85.1	7	14.9	47	0.129
≥ 3	126	74.6	43	25.4	169	

*BSA* body surface area, *BMI* body mass index, *DM* diabetes mellitus, *ECOG PS* Eastern Cooperative Oncology Group Performance Status, *WBC* white blood cell, *Hb* hemoglobin, *PLT* platelet, *CA19*–9 cancer antigen 19–9, *CVC*, central venous catheter

### Characteristics of venous thromboembolism

The characteristics of VTE are shown in Table 2. According to the site of VTE, VVT was the most common, occurring in 26 patients (51% of 51 VTE patients, 12% of all patients). Among all VTE patients, PE occurred in 15 (25.5%), and DVT occurred in 8 (13.7%). In terms of the time of VTE diagnosis, 23 patients (41.8% of 51 VTE patients and 10.6% of all patients) were included in the early VTE group. Meanwhile, the late VTE group included 28 patients (58.2% of 51 VTE patients and 13.0% of all patients). In both the early VTE and late VTE groups, VVT was the most common, followed by PE. Symptomatic VTE occurred in 15 patients (29.4% of VTE patients), whereas asymptomatic VTE was detected in 36 patients (70.6% of VTE patients). In symptomatic VTE, DVT was the most common, whereas VVT was the most common in asymptomatic VTE. Among the 51 VTE patients, anticoagulation treatment was administered to 15 patients (29.4%) using low-molecular-weight heparin, warfarin, and rivaroxaban. In the early VTE group, 9 patients (39.1%) received anticoagulation treatment and 6 (21.4%) received anticoagulation treatment in the late VTE group. In addition, among the 51 VTE patients, 32 patients (62.7%) continued chemotherapy after VTE diagnosis. Nineteen patients (37.3%) stopped chemotherapy and received supportive care because their general performance deteriorated simultaneously with VTE detection. Among the 19 patients who stopped chemotherapy, only 4 patients received anticoagulation treatment for a short period of approximately 2 weeks. These patients passed away within 6 weeks.

**Table 2:** Characteristics of venous thromboembolism in the study sample (*N* = 51)

	Early VTE	Late VTE	Total VTE	
	*N* (%, of all VTE)	*N* (%, of all VTE)	*N* (%, of all VTE)	% (of all patients)
Site of VTE:				
DVT	3 (5.9)	4 (7.8)	7 (13.7)	3.2
PE	5 (9.8)	8 (15.7)	13 (25.5)	6.0
VVT	12 (23.5)	14 (27.5)	26 (51)	12.0
PE + DVT	3 (5.9)	0 (0)	3 (5.9)	1.4
CVC related	0 (0)	2 (3.9)	2 (3.9)	0.9
Total	23 (45.1)	28 (54.9)	51 (100)	23.6
Symptoms:				
Symptomatic	7 (13.7)	8 (15.7)	15 (29.4)	6.9
Asymptomatic	16 (31.4)	20 (39.2)	36 (70.6)	16.7
Total	23 (45.1)	28 (54.9)	51 (100)	23.6
Coagulation				
Yes	9 (17.6)	6 (11.8)	15 (29.4)	6.9
No	14 (27.5)	22 (43.1)	36 (70.6)	16.7
Total	23 (45.1)	28 (54.9)	51 (100)	23.6
Time from the advanced pancreatic cancer to VTE diagnosis (months)				
Median (range)				2.2 (1.9–2.7)
Overall survival from VTE to death (months)				
Median (range)				2.4 (1.5–3.3)

*VTE* venous thromboembolism, *DVT* deep vein thrombosis, *PE* pulmonary embolism, *CI* cerebral infarction, *VVT* visceral venous thrombosis, *CVC* central venous catheter

### Survival and prognostic factors of all patients and patients with venous thromboembolism

The median OS of the 216 patients who received palliative chemotherapy was 6.2 months (95% confidence interval [CI] = 5.485–6.915), and the median OS of 51 patients with VTE who received palliative chemotherapy was 5.9 months (95% CI = 3.401–8.399). The median time from diagnosis of metastatic pancreatic cancer to VTE diagnosis was 2.2 months. In patients diagnosed with VTE, the median OS from the VTE diagnosis to death was only 2.4 months (95% CI = 1.5–3.3). VTE occurrence did not affect the duration of OS from the start of chemotherapy (*p* = 0.776). In addition, the presence of a central venous catheter and VTE-related symptoms or location of the VTE did not affect OS. However, a survival difference was observed based on the time of VTE diagnosis. In patients with early VTE, the median OS was significantly longer than in patients with late VTE or no VTE (*p* = 0.005) (Fig. 1a). The median OS of patients with early VTE was 3.7 months, however, the median OS of patients with late VTE was 9.8 months and that of patients without VTE was 6.3 months (*p* = 0.008) (Fig. 1b). In addition, the median progression-free survival (PFS) differed between the two groups. Patients with early VTE showed a significantly shorter PFS compared to patients with late VTE or no VTE (median PFS; 1.6 vs. 4.6 vs. 3.2 months, *p* < 0.001).

**Fig. 1:** Overall survival curves of all patients who received palliative chemotherapy according to venous thromboembolism occurrence. **a** Median OS of patents with early VTE was 3.7 months (95% CI, 2.135–5.265); that of patients with late VTE or without VTE was 6.4 months (95% CI, 5.522–7.278, *p* = 0.005). **b**Median OS of patents with early VTE was 3.7 months (95% CI, 2.135–5.265); that of patients with late VTE was 9.8 months (95% CI, 3.836–15.764) and that of patients without VTE was 6.3 months (95% CI, 5.493–7.107, *p* = 0.008).

The prognostic factors of all patients were investigated. To investigate of impact of VTE occurrence and other variables to OS, we analyzed using time-dependent multivariate Cox model. In that analysis, VTE occurrence itself did not show an association with poor OS (*p* = 0.711). However, early VTE *(p* = 0.001 for time of VTE occurrence) worse ECOG PS (2–3) (*p* = 0.004), higher NLR ≥2.7 *(p* = 0.048), low serum Na level < 135 mmol/L (*p* = 0.022), higher serum CA 19–9 level with < 1000 U/mL (*p* = 0.041), and presence of liver metastases (*p* = 0.046) were independent poor prognostic factors in multivariate Cox analysis (Table 3). Patients with early VTE had 1.897 times higher-risk of poor OS than patients with late VTE or no VTE (Table 3).

**Table 3:** Multivariate analysis of prognostic factors in all patients (*N* = 216)

	Overall survival (OS)		
	Hazard ratio	95% CI	*P-value*
Time of VTE occurrence (early vs. late and no VTE)	1.897	1.183–3.040	0.008
Khorana score (high-risk vs. intermediate-risk)	0.967	0.622–1.504	0.881
ECOG PS (2–3 vs 0–1)	2.118	1.267–3.541	0.004
NLR (≥2.7 vs. < 2.7)	1.432	1.003–2.046	0.048
PLR (≥180 vs. < 180)	1.257	0.884–1.787	0.202
WBC (≥11,000 /μLvs. <11,000 /μL)	1.29	0.788–2.113	0.311
Hb (< 10 g/dL vs. ≥10 g/dL)	1.242	0.760–2.030	0.387
Na (< 135 mmol/L vs. ≥135 mmol/L)	1.61	1.070–2.422	0.022
Albumin (< 3.5 g/dL vs. ≥3.5 g/dL)	1.036	0.691–1.552	0.865
CA19–9 (≥1000 U/mL vs. < 1000 U/mL)	1.364	1.013–1.836	0.041
Liver metastases (Yes vs. No)	1.382	1.006–1.899	0.046
Number of metastatic organs (≥3 vs. < 3)	0.752	.0521–1.086	0.129

*NLR* Neutrophil-to-lymphocyte ratio, *PLR* platelet-to-lymphocyte ratio, *Hb* hemoglobin, *CA19–9* cancer antigen 19–9, *WBC* White blood cell

The prognostic factors among patients diagnosed with VTE were investigated because these factors might be helpful to predict survival and to determine active treatment in this patient group. We found that early VTE (*p* = 0.001) was also an independent poor prognostic factor, as well as the number of metastatic organs ≥3 involved (*p* = 0.007) in patients with VTE. Among patients with VTE, those with early VTE had 3.768-fold higher risk of poor OS than those with late VTE (Table 4). Similar to the results for the entire patient group, other VTE-related factors including the Khorana score, VTE site, symptoms, and anticoagulant therapy were not statistically significant.

**Table 4:** Multivariate analysis of prognostic factors in patients with venous thromboembolism (*N* = 51)

	Overall survival (OS)		
	Hazard ratio	95% CI	*P-value*
Time of VTE occurrence (early vs. late)	3.768	1.705–8.328	0.001
Khorana score (high-risk vs. intermediate-risk)	1.005	0.454–2.224	0.990
Number of metastatic organs (≥3 vs. < 3)	5.961	1.640–21.665	0.007
Hb (< 10 g/dL vs. ≥10 g/dL)	1.277	0.344–4.739	0.714
Na (< 135 mmol/L vs. ≥135 mmol/L)	0.913	0.334–2.496	0.859
Albumin (< 3.5 g/dL vs. ≥3.5 g/dL)	1.605	0.482–5.343	0.441
CA 19–9 (≥1000 U/mL vs. < 1000 U/mL)	1.74	0.920–3.289	0.088
Lung metastases (Yes vs. No)	1.822	0.909–3.651	0.091

*NLR* neutrophil-to-lymphocyte ratio, *Hb* hemoglobin, *CA19–9* cancer antigen 19–9; *LN* lymph node

### Predictive factors associated with early venous thromboembolism diagnosis

Because the survival of patients with early VTE was significantly worse than that of patients without VTE or late VTE, the clinical characteristics of patients with early VTE and late VTE or no VTE were compared (Table 5). Age, sex, BSA, disease status, previous surgery, ECOG PS, CA 19–9 before chemotherapy, and number of metastatic organs did not show any differences between the two groups. However, the proportion of patients with serum Na level < 135 mmol/L was higher in patients with early VTE (*p* = 0.008). Among the variables included in the Khorana’s prediction model, high PLT counts (≥350,000/μL) were observed in a higher proportion of patients with early VTE (*p* = 0.008). In addition, the proportion of patients in the high-risk group (Khorana score ≥ 3) was higher in the early VTE group (*p* = 0.014). Multivariate analysis using a logistic regression model showed that classification into the high-risk group, with Khorana score ≥ 3 and hyponatremia with serum Na levels < 135 mmol/L was strongly associated with the occurrence of synchronous VTE (odds ratio [OR] 5.109; 95% CI = 1.010–25.845; *p* = 0.049 for Khorana score, OR 10.304; 95% CI = 1.036–102.466; *p* = 0.047 for hyponatremia).

**Table 5:** Factors associated with early venous thromboembolism (N = 216)

	No or late VTE		Early VTE		Total	*P-value*
	N	%	N	%	N	
Age						
< 70	131	87.3	19	12.7	150	0.147
≥ 70	62	93.9	4	3.1	66	
Sex						
Male	121	92.4	10	7.6	131	0.075
Female	72	84.7	13	15.3	85	
BSA						
< 1.8	177	90.3	19	9.7	196	0.155
≥ 1.8	16	80	4	20	20	
BMI						
< 30 kg/m^2^	188	89.5	22	10.5	210	0.628
≥ 30 kg/m^2^	5	83.3	1	16.7	6	
DM						
No	106	86.2	23	17	123	0.082
Yes	87	93.5	6	6.5	93	
Site of primary mass						
Head	89	88.1	12	11.9	101	0.261
Body	34	97.1	1	2.9	35	
Tail	70	87.5	10	12.5	80	
Previous surgery						
Palliative	11	91.7	1	8.3	12	0.789
None	182	89.2	22	10.8	204	
ECOG PS						
0–1	174	88.8	22	11.2	196	0.390
2–3	19	95	1	5	20	
WBC						
< 11,000/μL	162	89.5	19	10.5	181	0.87
≥ 11,000/μL	31	88.6	4	11.4	35	
Hb						
< 10 g/dL	28	84.8	5	15.2	33	0.276
≥ 10 g/dL	165	90.2	18	9.8	183	
Platelet						
< 350,000/μL	172	91.5	16	8.5	188	0.008
≥ 350,000/μL	21	75	7	25	28	
Khorana score						
Intermediate-risk (2)	126	93.3	9	6.7	135	0.014
High-risk (≥3)	67	82.7	14	17.3	81	
Na						
< 135 mmol/L	26	76.5	8	23.5	34	0.008
≥ 135 mmol/L	167	91.8	15	8.2	182	
CA19–9						
< 1000 U/mL	105	89.7	12	10.3	117	0.839
≥ 1000 U/mL	88	88.9	11	11.1	99	
Number of metastatic organs						
< 3	45	95.7	2	4.3	47	0.108
≥ 3	148	87.6	21	12.4	169	

*BSA* body surface area, *BMI* body mass index, *DM* diabetes mellitus, *ECOG PS* Eastern Cooperative Oncology Group Performance Status, *WBC* white blood cell, *Hb* Hemoglobin, *PLT* platelet, *CA19–9* cancer antigen 19–9

## Discussion

VTE is a common complication of pancreatic cancer. However, data regarding the incidence, characteristics, or survival of patients with metastatic pancreatic cancer with VTE who receive palliative chemotherapy are limited. In the present study, the incidence of VTE was 23.6%, which was similar to that of previous reports. A randomized controlled study of patients with pancreatic cancer receiving chemotherapy performed to assess the value of simultaneous thromboprophylaxis with chemotherapy found that VTE incidence during the trial in the no thromboprophylaxis group was 28% [10]. In another retrospective study, the incidence of VTE in patients with pancreatic cancer receiving chemotherapy was 35.7% [11]. In the present study, we found that VTE occurrence itself did not affect the survival of patients with metastatic pancreatic cancer receiving palliative chemotherapy. In general, VTE occurrence is known to lead to poor survival outcomes in patients with cancer. In contrast, some studies have reported that VTE occurrence in patients with pancreatic cancer was not associated with poor survival, which is similar to the results of our study [12, 13]. Furthermore, the most important VTE related prognostic factor in the present analysis was the time of VTE diagnosis, rather than the occurrence of VTE. Patients diagnosed with VTE around the initiation of cancer chemotherapy, defined as early VTE, showed significantly poor survival in this study. The prognosis was even worse in patients with early VTE among the subgroup of patients with VTE, resulting in an almost 4-fold increased risk of death. Nonetheless, most previous studies regarding VTE focused on all VTE events during treatment courses; only one study investigated early VTE in patients with pancreatic cancer receiving chemotherapy. In the study by Mandala et al. comprising 227 patients with nonresectable pancreatic cancer, the incidence of early VTE was 12.3%, [14], which was similar to 10.6% of the 216 included patients in our study. Although early VTE did not affect the PFS or OS on multivariate analysis in the study of Mandala et al., it was associated with poor response to chemotherapy.

VTE development in patients with cancer results from multifactorial mechanisms. The main pathogenesis is associated with the generation of both intrinsic and extrinsic hypercoagulable status owing to cancer cells. Cancer cells stimulate the coagulation cascade by increasing the production of procoagulant activators such as tissue factor (TF) [15]. The upregulated coagulation cascade affects not only systemic coagulation but also tumor growth and metastasis through activation of angiogenesis signaling pathways [16]. This stimulation of tumor angiogenesis leads to more aggressive tumor progression. A study on pancreatic cancer found that TF is also expressed in pancreatic cancer cells and its expression was associated with poor histologic grade and worse prognosis [17]. Moreover, the expression of TF on tumor cells resulted in increased mitogenic activity through enhanced vascular permeability and synthesis of vascular endothelial cell growth factor [18]. Therefore, our analysis suggests that the occurrence of early VTE at the time of cancer diagnosis indicates an enhanced angiogenic condition of the tumor that implies biologically more aggressive characteristics at baseline, thus possibly resulting in poor OS. In addition, a hypercoagulable status has been associated with poor response to chemotherapy [19]. Moreover, additive morbidity owing to VTE and interruption or delay of chemotherapy due to VTE management or anticoagulation treatment may also be associated with poor survival in patients with early VTE.

In addition, a higher number of metastatic organs were also a significant poor prognostic factor among patients with VTE in the present study. High numbers of metastatic organs are associated with a relatively large tumor burden and advanced tumor status, factors that cause poor survival outcome. In previous analyses that included patients with pancreatic cancer from resectable stage to advanced disease, patients with metastatic disease showed a higher risk of death compared to other patients, when they were diagnosed with VTE [12]. Even in the present study, which included only patients with advanced stage pancreatic cancer, patients with a higher number of metastatic organs showed significantly worse prognosis among patients with VTE. Therefore, we should focus on this subgroup of patients with poor prognostic factors to improve survival outcomes. For example, further investigation on the effectiveness of anticoagulation treatment in patients with a higher tumor burden and/or who experience early VTE are necessary. VTE-related prognostic factors in this study might be helpful to select patients for future clinical trials.

Prediction of VTE is important because it encourages greater attention to the occurrence of VTE in patients presenting significant risk factors. In the present study, we focused on investigating the predictors of early VTE because it was a significant poor prognostic VTE-related factor. Among all patients, those with a PLT count > 350,000/μL, which is a factor included in Khorana’s model, showed a higher incidence of VTE. Increased PLT count is associated with hyperviscosity and has been associated with increased risk of VTE in a previous study [20]. Unexpectedly, a serum Na level < 135/mmol was a significant risk factor for occurrence of early VTE in this study. Hyponatremia is not a well-known predictive factor for VTE, but some studies have reported the association of VTE and hyponatremia. In a study of Chinese non-small cell lung cancer patients, the risk of VTE was increased in patients with hyponatremia (< 130/mmol) [21]. In addition, in a study of pediatric patients who underwent orthopedic surgery, hyponatremia was reported as a risk factor for VTE [22]. Nevertheless, the mechanism underlying the association between hyponatremia and early VTE is difficult to explain; however, hyponatremia prior to chemotherapy may reflect poor oral intake or a poor general medical status of the patient, and this state may be associated with a thrombosis-prone condition. Further studies are needed to investigate the mechanisms involved.

In the present study, classification into the high-risk group defined using Khorana’s model was also an important predictive marker of early VTE. No difference was observed in the incidence of all VTE between the intermediate- and high-risk groups defined according to Khorana’s model; however, a significant difference for the risk of early VTE occurrence was observed. The initial study used to define Khorana’s prediction model included patients with various types of cancer [4]. Only 54 (2.0%) gastric and 19 (1.4%) pancreatic cancer patients were included in the derivation cohort and the validation cohort of that study. Even in other studies for external validation, the number of patients with pancreatic cancer was small [23, 24]. In addition, according to previous studies, which included only patients with pancreatic cancer, conflicting findings were observed regarding the predictive role of the model. Munoz Martin et al. compared the incidence of VTE detected within 6 months after diagnosis between high- and intermediate-risk groups according to Khorana’s model in 84 patients with pancreatic cancer receiving chemotherapy. VTE incidence was higher in the high-risk group (37.5%) than in the intermediate-risk group (33.3%) [11]. Conversely, van Es et al. reported that Khorana’s model did not discriminate between intermediate risk and high risk of VTE because VTE incidence did not differ between the two groups in their study that included 178 patients with pancreatic cancer receiving chemotherapy [25]. However, we can suggest that Khorana’s model has a predictive role particularly for early VTE in patients with pancreatic cancer receiving chemotherapy and our study has value in the validation of the model that included 216 patients, which is by far the greatest number of patients with same disease status included in comparable studies.

In the present study, symptomatic VTE occurred in 6.9% of patients. In general, symptomatic VTE has received greater attention because it can negatively impact on quality of life, delay cancer treatment, and result in additive anticoagulation treatment. In contrast, asymptomatic VTE has not been a subject of common interest in this field. Nevertheless, symptomatic VTE did not affect OS in the present study. Moreover, two-thirds of patients with early VTE exhibited asymptomatic VTE. Therefore, we suggest that the occurrence and detection time of VTE is more important, regardless of the presence of symptoms; VTE screening at the start of palliative chemotherapy should be performed even in patients with no VTE-related symptoms. Some VTEs, such as PE or VVT, can be detected despite the absence of symptoms because patients are required to undergo imaging analysis including chest and abdominopelvic CT to assess their cancer status prior to the initiation of chemotherapy. In addition, laboratory analysis using D-dimer, which is a fibrin degradation product and reflects the activation of hemostasis and fibrinolysis, would be helpful because D-dimer is a well-known and widely available biomarker for screening of VTE in the general population and in some cancer patients [26]. However, the potential use of D-dimer as a predictive factor for VTE in patients with pancreatic cancer receiving palliative chemotherapy has not been reported and further investigation is necessary. Because concordant markers are yet to be confirmed in clinical practice, focusing on the Khorana score, which has been shown to have meaningful significance in predicting the occurrence of VTE, could be helpful, particularly in predicting synchronous VTE, as in our study. Further research regarding the use of coagulation-related markers and clinical factors would be helpful for screening for VTE located outside of the routine CT imaging field or for those with microcoagulable status barely detectable using imaging modalities.

This study is limited by its single institution retrospective design. We could not analyze the association or role of clinical factors with VTE-related or coagulation-related laboratory tests because of insufficient data. We only determined an association of clinical factors and VTE. However, this study has value because of the higher number of patients included compared to other previous studies with a similar objective. The present study should provide the basis for further investigations, such as studies into the role of anticoagulation therapy for patients with pancreatic cancer and early VTE.

## Conclusions

In conclusion, early occurrence and detection of VTE at the beginning of palliative chemotherapy is an important poor prognostic factor for patients with metastatic pancreatic cancer and the Khorana score and serum Na levels are valuable for predicting the occurrence of early VTE in these patients. Clinicians should be particularly attentive to patients with pancreatic cancer with high Khorana scores and low serum Na and the occurrence of VTE around the start of chemotherapy. Furthermore, future research to improve survival outcomes for patients who have poor prognostic factors is desperately needed.

## Abbreviations

BMI: Body mass index
BSA: Body surface area
CI: Confidence interval
CT: Computed tomography
DM: Diabetes mellitus
DVT: Deep vein thrombosis
ECOG PS: Eastern Cooperative Oncology Group Performance Status
Hb: Hemoglobin
MRI: Magnetic resonance imaging
NLR: Neutrophil-to-lymphocyte ratio
OR: Odds ratio
OS: Overall survival
PE: Pulmonary embolism
PLR: Platelet-to-lymphocyte ratio
PLT: Platelet
VTE: Venous thromboembolism
VVT: Visceral venous thrombosis
WBC: White blood cell
